RETRACTED

# *In vitro* antioxidant and anticancer activity of young *Zingiber officinale *against human breast carcinoma cell lines

**DOI:** 10.1186/1472-6882-11-76

**Published:** 2011-09-20

**Authors:** Shahedur Rahman, Faizus Salehin, Asif Iqbal

**Affiliations:** 1 Department of Biotechnology and Genetic Engineering, Islamic University, Kushtia-7003, Bangladesh; 2 Department of Biotechnology and Genetic Engineering, University of Development Alternative, Dhaka, Bangladesh

## Abstract

**Background:**

Ginger is one of the most important spice crops and traditionally has been used as medicinal plant in Bangladesh. The present work is aimed to find out antioxidant and anticancer activities of two Bangladeshi ginger varieties (Fulbaria and Syedpuri) at young age grown under ambient (400 μmol/mol) and elevated (800 μmol/mol) CO_2 _concentrations against two human breast cancer cell lines (MCF-7 and MDA-MB-231).

**Methods:**

The effects of ginger on MCF-7 and MDA-MB-231 cell lines were determined using TBA (thiobarbituric acid) and MTT [3-(4,5-dimethylthiazolyl)-2,5-diphenyl-tetrazolium bromide] assays. Reversed-phase HPLC was used to assay flavonoids composition among Fulbaria and Syedpuri ginger varieties grown under increasing CO_2 _concentration from 400 to 800 μmol/mol.

**Results:**

Antioxidant activities in both varieties found increased significantly (P ≤ 0.05) with increasing CO_2 _concentration from 400 to 800 μmol/mol. High antioxidant activities were observed in the rhizomes of Syedpuri grown under elevated CO_2 _concentration. The results showed that enriched ginger extract (rhizomes) exhibited the highest anticancer activity on MCF-7 cancer cells with IC_50 _values of 34.8 and 25.7 μg/ml for Fulbaria and Syedpuri respectively. IC_50 _values for MDA-MB-231 exhibition were 32.53 and 30.20 μg/ml for rhizomes extract of Fulbaria and Syedpuri accordingly.

**Conclusions:**

Fulbaria and Syedpuri possess antioxidant and anticancer properties especially when grown under elevated CO_2 _concentration. The use of ginger grown under elevated CO_2 _concentration may have potential in the treatment and prevention of cancer.

## Background

Cancer is a multi-step disease incorporating physical, environmental, metabolic, chemical and genetic factors, which play a direct and/or indirect role in the induction and deterioration of cancers. Diet containing antioxidant rich fruits and vegetables significantly reduces the risk of many cancer diseases suggesting that antioxidants could be effective agents for the inhibition of cancer spread. These agents are present in the diet as a group of compounds with low toxicity, safe and generally accepted [1]. The Isolated polyphenols from different plants have been considered as indicator in a number of cancer cell lines at different evolutionary stages of cancer. Anticancer activities of Flavonoids were described in various studies [2]. Some tests showed antitumor properties of quercetin including the inhibition of cancer cell proliferation and migration [3]. The isolated polyphenols from strawberry including kaempferol, quercetin, anthocyanins, coumaric acid and ellagic acid were shown to inhibit the growth of human cancer cell lines originated from breast (MCF-7), oral (KB, CAL-27), colon (HT-29, HCT-116), and prostate (LNCaP, DU-145) [4]. Similar results have also been reported in other studies with wine extracts, isolated polyphenols (resveratrol, quercetin, catechin, and epicatechin) and green tea polyphenols (epigallocatechin, epicatechin) [5,6]. Arts *et al. *reported of catechin's ability to control postmenopausal cancer in woman [7]. They found that catechin intake may prevent rectal cancer. Epicatechin and gallocatechin-3-gallate induce reduction in experimental lung tumour metastasis (77% and 46%). Epigallocatechin-3-gallate is an effective antiangiogenesis agent, which inhibits tumour cell invasion and proliferation [8]. It also inhibits the growth of the NBT-II bladder tumour cells and breast cancer cell lines [9]. Manthey *et al. *reported that citrus flavonoids inhibited the growth of HL-60 leukaemia cells [10]. Kaempferol belongs to the flavonoids group. Luo *et al. *showed kaempferol inhibited the growth of ovarian cancer cell lines (91%) and A2780/CP70 (94%) by concentration of 20 μM and 40 μM respectively [11]. Inhibition of breast cancer cell lines (MCF-7 and MDA-MB-231) by quercetin was reported by Gibellini *et al. *[12]. In recent years, researches about anticarcinogenic potential of quercetin have exhibited its promise as an anticancer agent. Likewise, *in vitro *and *in vivo *studies showed that quercetin was able to inhibit viability of leukemic cells, colon and ovarian carcinoma cells, and especially human breast cancer cells.

RETRACTED

The Zingiberaceae family is well-known in Southeast Asia and many of its species are being used as traditional medicine, which is found to be effective in the treatment of several diseases. *Zingiber officinale *is generally used as a culinary spice in Bangladesh and as well as for the treatment of oral diseases, leucorrhoea, stomach pain, stomach discomfort, diuretic, inflammation and dysentery. Shukla *et al. *reported cancer preventive properties of ginger and showed that this ability is related to flavonoid and polyphenolic components of fresh ginger extract especially quercetin [13]. Kuokkanen *et al. *showed that the concentration of total phenolics was significantly increased in the birch leaves produced in the CO_2_-enriched air, as has also been observed in the experiments of Ibrahim *et al. *[14,15]. Emerging management strategies are using eco-physiological factors to elevate phytochemical concentrations in food crops. Some eco-physiological conditions that are thought to have significant impact on the enhancement of health-promoting phytochemicals in a number of plants include environmental conditions, cultural and management practices [16]. In addition, there is an increasing interest in using appropriate strategies of management practices to improve the quality of food crops by enhancing their nutritive and health-promoting properties. The results of previous studies indicated that the synthesis of phenolics and flavonoids in ginger can be increased and affected by using CO_2 _enrichment and following that, the antioxidant activity in young ginger extracts could also be improved [17]. Information about anticancer and antioxidant activities of enriched ginger by elevated CO_2 _concentration is scarce. On the other hand, the impacts of cultural conditions and CO_2 _concentration on biopharmaceutical production in herbs have not been widely investigated and it is needed to be understood, especially when the objective is the optimization of the herb chemistry. In this study, we aimed to explore antioxidant potential and anticancer activities of two Bangladeshi ginger varieties (*Zingiber officinale*) at young age and grown under different CO_2 _concentration.

## Methods

### Plant material

Two varieties of *Zingiber officinale *Roscoe (Fulbaria and Syedpuri) rhizomes were germinated for two and half weeks and then transferred to polyethylene bags which were filled with soilless mixture of burnt rice husk and coco peat in a ratio 1:1. After two and half weeks, those plants were transferred to CO_2 _growth chamber with two different CO_2 _concentrations (400 μmol/mol, ambient; 800 μmol/mol, elevated CO_2 _concentration). Pure carbon dioxide (99.6% purity) was supplied from high pressure carbon dioxide cylinder and injected through a pressure regulator into the growth chamber. Irradiance, relative humidity and air temperature of chamber were controlled using integrated control, monitoring and data management system software. Plants were harvested at 15 weeks and aerial parts and rhizomes separated and freeze dried and kept in -90°C for future analysis.

### Extract preparation

Aerial parts and rhizomes were dried (freeze dry) to constant weights. Aerial parts and rhizomes (1 g) were powdered and extracted using methanol (50 ml), with continuous swirl for 1 h at room temperature using an orbital shaker. Extracts were filtered under suction, evaporated and crude extract stored at -25°C. These crude extracts were used in this study [18].

RETRACTED

### Determination of antioxidant activity

#### TBA assay

The method of Ottolenghi (1959) was used to determine the TBA (thiobarbituric acid) values of the samples [19]. The formation of malonaldehyde is the basis for the well-known TBA method used for evaluating the extent of lipid peroxidation. At low pH and high temperature (100°C), malonaldehyde binds TBA to form a red complex that can be measured at 532 nm. The increase amount of the red pigment formed correlates with the oxidative rancidity of the lipid. 2 ml of 20% trichloroacetic acid (CCI_3_COOH) and 2 ml TBA aqueous solution were added to 1 ml of sample solution and incubated. The mixture was then placed in a boiling water bath for 10 min. After cooling, it was centrifuged at 3,000 rpm for 20 min and the absorbance of the supernatant was measured at 532 nm. Antioxidant activity was determined based on the absorbance.

#### Cell culture and treatment

Human breast cancer cell lines (MCF-7 and MDA-MB-231) were obtained from the American Tissue Culture Collection (ATCC) (Rockville, MD) and were cultured in 100 μl of Roswell Park Memorial Institute medium (RPMI) 1640 media supplemented with 10% fetal bovine serum (FBS), 100 U/ml penicillin and 100 μg/ml streptomycin. MCF-7 and MDA-MB-231 cells were incubated overnight at 37°C in 5% CO_2 _for cells attachment [20].

Both non invasive MCF-7 and highly invasive MDA-MB231 cancer cells were used in this study to verify the effectiveness of ginger extract against them.

### Determination of anticancer activity

#### MTT assay

The assay detects the reduction of MTT [3-(4, 5-dimethylthiazolyl)-2, 5-diphenyl-tetrazolium bromide] by mitochondrial dehydrogenase to blue formazan product, which reflects the normal functioning of mitochondria and hence the cell viability. The experiment was conducted as described by Mosmann (1983) [21]. Briefly, the cancer cells were seeded in 96-well plates at a density of 1 × 10^4 ^cells/well in 100 μl RPMI. After twenty-four hours of seeding, the medium was removed and then the cells were incubated for 3 days with RPMI with the absence and/or the presence of various concentration of ginger extracts. Ginger extract was added at various concentrations ranging from 4.6, 9.3, 18.7, 37.5, 75, 150 and 300 μg/ml. After incubation, 20 μl of MTT reagent was added into each well. These plates were incubated again for 4 h in CO_2 _incubator at 37°C. The resulting MTT-products were determined by measuring the absorbance at 570 nm using ELISA reader [22]. The cell viability was determined using the formula:

Viability %=(optical density of sample∕optical density of control)×100

IC_50 _values were calculated as the concentrations that show 50% inhibition of proliferation on any tested cell line.

RETRACTED

Same batch of ginger extracts were used for both TBA and MTT assay.

### High performance liquid chromatography (HPLC)

#### Flavonoid extract preparation

Aliquots of aerial parts and rhizomes (0.25 g) were extracted with 60% aqueous methanol (20 ml). 6 M HCl (5 ml) was added to each extract to give a 25 ml solution of 1.2 M HCl in 50% aqueous methanol. Extracts were refluxed at 90°C for 2 h. Extract aliquots of 500 μl, taken both before and after hydrolysis, were filtered through a 0.45 μm filter [23].

#### Analysis of flavonoids composition

Reversed-phase HPLC was used to assay flavonoid compositions. The Agilent HPLC system used consisted of a model 1100 pump equipped with a multi-solvent delivery system and an L-7400 ultraviolet (UV) detector. The column was an Agilent C18 (5 μm, 4.0 mm internal diameter 250 mm). The mobile phase composed of: (A) 2% acetic acid (CH_3_COOH) and (B) 0.5% acetic acid-acetonitrile (CH_3_CN), (50:50 v/v), and gradient elution was performed as follows: 0 min, 95:5; 10 min, 90:10; 40 min, 60:40; 55 min, 45:55; 60 min, 20:80 and 65 min, 0:100. The mobile phase was filtered under vacuum through a 0.45 μm membrane filter before use. The flow rate was 1 ml/min and UV absorbance was measured at 280-365 nm. The operating temperature was maintained at room temperature [24]. Identification of the flavonoids was achieved by comparison with retention times of standards, UV spectra and calculation of UV absorbance ratios after coinjection of samples and standards [25].

### Statistical analysis

The experimental results were expressed as mean ± standard deviation of three replicates. Where applicable, the data were subjected to one-way analysis of variance (ANOVA) and the differences among samples were determined by Duncan's Multiple Range Test using the SPSS v14 and MSTATC programs. P-value of ≤ 0.05 was regarded as significant.

## Results and discussion

### Antioxidant activity

The results obtained from the preliminary analysis of antioxidant activity are shown in Table 1. According to the data obtained significant differences were observed among treatments for antioxidant activities. From the result, the antioxidant activity of aerial parts was higher than rhizomes extracts in both varieties that were grown under ambient CO_2 _concentration. The results also had indicated that antioxidant activities increased significantly by elevated CO_2 _concentration. Antioxidant activity was enhanced in rhizomes by elevated CO_2 _concentration more than in aerial parts with highest value of TBA (77.98%) were obtained from Syedpuri rhizomes. The aerial parts extract of Fulbaria and Syedpuri in ambient and elevated CO_2 _condition exhibited strong potential of free radical scavenging activity. According to the results, TBA content of the Syedpuri aerial parts grown in ambient CO_2 _concentration reached to 70.59%, while at the same extract concentration, that of the rhizomes was 67.79%. In ambient CO_2 _concentration, differences between aerial parts and rhizomes in both varieties for TBA activity was not significant, while in elevated CO_2 _concentration significant differences was observed between different parts of each variety. Many researchers had shown that high total flavonoids content increases antioxidant activity and there was a linear correlation between flavonoids content and antioxidant activity [18,26].

RETRACTED

**Table 1:** Antioxidant activity of *Zingiber officinale *extracts grown under different CO_2 _concentrations (measured by the TBA method)

CO_2 _(μmol/mol)	Varieties	Parts	TBA
	Fulbaria	Aerial parts Rhizomes	69.29 ± 2.32^c,d^ 67.93 ± 1.81^d^
400			
	Syedpuri	Aerial parts Rhizomes	70.59 ± 1.89^a,c,d^ 67.79 ± 0.64^d^

	Fulbaria	Aerial parts Rhizomes	71.01 ± 2.52^a,c^ 75.05 ± 1.63^b,e^
800			
	Syedpuri	Aerial parts Rhizomes	73.78 ± 1.21^a,e^ 77.98 ± 1.20^b^

All analyses are the mean of triplicate measurements ± standard deviation. Means not sharing a common letter were significantly different at P < 0.05.

Results expressed in percent.

### Anticancer activity

As shown in Table 2, parts (aerial parts and rhizomes) of two ginger varieties were found to express MCF-7 and MDA-MB-231 cancer cell inhibitory activity when tested at concentrations of 4.6-300 μg/ml. At a concentration of 37.5 μg/ml, though, most of the extracts exhibited strong anticancer activity towards MCF-7 and MDA-MB-231 cells, at this concentration, extract of Syedpuri rhizomes grown under elevated CO_2 _concentration exhibit lowest MCF-7 and MDA-MB-231 cell viability at 39.01% and 40.16% respectively. Moreover, MCF-7 and MDA-MB-231 treated with tamoxifen (positive control) showed 24.9% and 26.7% viability in same concentration (37.5 μg/ml). In contrast, for MCF-7 cell, the anticancer activity of aerial parts extract in ambient and elevated CO_2 _concentration was significantly stronger than that of the rhizomes extract especially in Syedpuri variety. In addition, for MDA-MB-231 cell, the anticancer activity of aerial parts extract in ambient CO_2 _concentration was significantly stronger than that of the rhizomes extracts, but, with increasing of CO_2 _concentration anticancer power increased significantly in rhizomes of both varieties. However, of all extracts investigated, Syedpuri rhizomes that were obtained from plants grown under elevated CO_2 _concentration exhibited the strongest anticancer activities towards cancer cells. The IC_50 _values for MCF-7 and MDA-MB-231 cells were 25.7 and 30.2 μg/ml respectively (Table 3). While IC50 value of rhizomes extract of Syedpuri grown in ambient CO_2 _for MCF-7 and MDA-MB-231 cells were 47 and 38.8 μg/ml accordingly. However, with the increase of CO_2 _concentration, IC_50 _value decreased significantly in both varieties. Furthermore, IC_50 _values of tamoxifen as a positive control for MCF-7 and MDA-MB-231 cells were 19.7 and 22.89 μg/ml respectively.

RETRACTED

**Table 2:** Anticancer activities of *Zingiber officinale *extracts against MCF-7 and MDA-MB-231 cell lines (determined by the MTT assay at concentration 37.5 μg/ml)

CO_2 _(μmol/mol)	Varieties	Parts	MCF-7	MDA-MB-231
	Fulbaria	Aerial parts Rhizomes	59.65 ± 2.55^b^ 57.56 ± 1.68^b^	63.31 ± 1.85^e^ 69.41 ± 2.30^b^
400				
	Syedpuri	Aerial parts Rhizomes	50.65 ± 0.56^e^ 56.98 ± 1.74^b^	58.12 ± 1.09^a^ 66.61 ± 2.31^b,e^

	Fulbaria	Aerial parts Rhizomes	40.37 ± 1.46^c^ 48.97 ± 1.04^e^	48.16 ± 1.03^c^ 44.35 ± 1.86^d^
800				
	Syedpuri	Aerial parts Rhizomes	44.93 ± 1.53^a^ 39.01 ± 2.1^c^	43.02 ± 1.99^d^ 40.16 ± 2.42^f^

Positive control	Tamoxifen		24.9 ± 1.6	26.70 ± 2.11

All analyses are the mean of triplicate measurements ± standard deviation. Means not sharing a common letter were significantly different at P ≤ 0.05.

Results expressed in percent of cell viability.

**Table 3:** IC_50 _values of *Zingiber officinale *extracts against MCF-7 and MDA-MB-231 cancer cell lines (expressed in μg/ml)

CO_2 _(μmol/mol)	Varieties	Parts	MCF-7	MDA-MB-231
	Fulbaria	Aerial parts Rhizomes	51.39 ± 1.32^b^ 52.01 ± 2.11^b^	56.12 ± 2.15^e^ 62.81 ± 1.60^b^
400				
	Syedpuri	Aerial parts Rhizomes	36.80 ± 1.32^a^ 47.00 ± 1.16^e^	46.87 ± 0.45^a^ 38.80 ± 1.81^c^

	Fulbaria	Aerial parts Rhizomes	29.83 ± 1.37^c^ 34.80 ± 1.80^a^	34.60 ± 2.16^d^ 32.53 ± 1.07^d^
800				
	Syedpuri	Aerial parts Rhizomes	27.21 ± 2.01^d^ 25.70 ± 0.64^f^	32.85 ± 0.89^d^ 30.20 ± 0.81^f^

All analyses are the mean of triplicate measurements ± standard deviation.

Means not sharing a common letter were significantly different at P ≤ 0.05.

### HPLC analysis of flavonoids

The results obtained from the preliminary analysis of flavonoids are shown in Table 4. Increasing the CO_2 _concentration from 400 to 800 μmol/mol resulted in enhanced quercetin, catechin, kaempferol and fisetin levels in the aerial parts and rhizomes of both varieties. On the other hand, the contents of epicatechin and morin decreased in ginger parts with rising of CO_2 _concentration from ambient to 800 μmol/mol. Some study results indicated that increasing the CO_2 _concentration from 400 to 800 μmol/mol resulted in enhanced quercetin, catechin, kaempferol and fisetin levels in the aerial parts and rhizomes of *Zingiber officinale *varieties and following that, the antioxidant activity in young ginger extracts could also be improved [25]. Findings of this current study supported previous researcher's findings and showed that anticancer effect of ginger extracts increase with increasing CO_2 _concentration.

RETRACTED

**Table 4:** The concentrations of some flavonoids compounds in two varieties of *Zingiber officinale*, Fulbaria and Syedpuri grown under various CO_2 _concentrations

	Fulbaria				Syedpuri			
	
Flavonoid compounds	400		800		400		800	
	
	Aerial parts	Rhizomes	Aerial parts	Rhizomes	Aerial parts	Rhizomes	Aerial parts	Rhizomes
Quercetin	0.961 ± 0.013^a^	0.894 ± 0.039^a^	1.22 ± 0.06^e^	1.137 ± 0.023^e^	1.19 ± 0.122^b,e^	0.985 ± 0.032^a^	1.33 ± 0.124^b^	1.26 ± 0.01^b^
Epicatechin	0.128 ± 0.028^b^	0.085 ± 0.007^a,e^	0.073 ± 0.009^a^	0.049 ± 0.018^c^	0.12 ± 0.004^b^	0.103 ± 0.0034^d,e^	0.096 ± 0.021^a,e^	0.038 ± 0.009^c^
Catechin	0.416 ± 0.024^c^	0.492 ± 0.020^a,c^	0.673 ± 0.044^b,e^	0.637 ± 0.044^e^	0.668 ± 0.079^b,e^	0.533 ± 0.034^a^	0.734 ± 0.014^b^	0.684 ± 0.05^b,e^
Kaempferol	0.041 ± 0.006^d^	0.052 ± 0.003^c,d^	0.117 ± 0.014^a^	0.147 ± 0.023^e^	0.051 ± 0.002d^d^	0.067 ± 0.005^c^	0.162 ± 0.011^b,e^	0.184 ± 0.019^b^
Fisetin	0.982 ± 0.022^d^	0.633 ± 0.033^f^	2.051 ± 0.27^a^	2.88 ± 0.19^b^	1.53 ± 0.121^c^	1.32 ± 0.13^c^	2.37 ± 0.397^e^	3.12 ± 0.185^b^
Morin	0.532 ± 0.057^d^	0.464 ± 0.014^d^	0.491 ± 0.052^d^	0.876 ± 0.046^b^	0.765 ± 0.024^e^	0.607 ± 0.006^c^	0.662 ± 0.029^a^	0.517 ± 0.025^d^

All analyses are the mean of triplicate measurements ± standard deviation.

Means not sharing a common letter were significantly different at P ≤ 0.05.

Results expressed in mg/g of dry plant material.

Flavonoids are among the best candidates for mediating the protective effect of diets which are found in fruits and vegetables with respect to colorectal cancer. Study shows relative activity being as quercetin > apigenin > fisetin> kaempferol. Quercetin belongs to the flavonoids group due to its powerful antioxidant activity. Previous studies showed that quercetin may help to prevent cancer, especially prostate cancer [27]. Scambia *et al. *reported quercetin inhibited human breast cancer cells (MCF-7 and MDA-MB231) significantly [28]. Du *et al. *explained mechanism of breast cancer inhibition by quercetin [29]. In ginger quercetin is abundant flavonoid compound [25,26,30]. Antioxidant activity of quercetin was believed to have cytoprotective role against oxidative stress. It seemed that quercetin not only protects cells from free radical damage through antioxidant effect, but also motivates apoptotic cell death via pro-oxidant activity and inhibits tumourigenesis. Hence, anticancer power maybe related to quercetin content in those varieties. In addition, flavonoid compounds could probably be responsible for the anticancer activity of *Zingiber officinale*. Further research is required to untangle the specific bioactive compounds responsible for the anticancer properties of the extracts of *Zingiber officinale *varieties.

RETRACTED

## Conclusions

Currently, about 50% of drugs used in clinical trials for anticancer activity were isolated from natural sources such as herbs and spices or related to them [31]. A number of active compounds such as flavonoids, diterpenoids, triterpenoids and alkaloids have been shown to possess anticancer activity. According to the report of the American National Cancer Institute (NCI), the criterion of anticancer activity for the crude extracts of herbs is an IC50<30 μg/ml [32]. Thus, according to the results from current study seems that enriched ginger varieties developed by elevated CO_2 _concentration could be employed in ethno-medicine in the treatment of cancerous diseases.

There are some limitations of this study. Relationship between flavonoids concentration and antioxidant activity were not determined. Moreover, only cytotoxicity was determined but apoptosis and cell cycle analysis were not performed.

Our results in this study indicate that some compounds in Bangladeshi ginger varieties at young age possess anticancer activities and may contribute in the therapeutic effect of this medicinal herb. However, there is a need of detailed scientific study on traditional medical practices to ensure that valuable therapeutic knowledge of some plants is preserved and also to provide scientific evidence for their efficacies.

## Competing interests

The authors declare that they have no competing interests.

## Authors' contributions

SR and FS participated in the design, coordinating and carried out the study and also drafted the manuscript. AI performed the statistical analysis. All authors read and approved the final manuscript.

## Pre-publication history

The pre-publication history for this paper can be accessed here:

http://www.biomedcentral.com/1472-6882/11/76/prepub
